# Correlation between Parturients' Uterine Artery Blood Flow Spectra in the First and Second Trimesters of Pregnancy and Fetal Growth Restriction

**DOI:** 10.1155/2021/2129201

**Published:** 2021-12-14

**Authors:** Hongna Yu, Meiqin Yuan, Ling Wang, Xia Li, Meiping Jiang

**Affiliations:** Department of Ultrasound, Yantai Yuhuangding Hospital, Yantai, 264000, Shandong Province, China

## Abstract

**Objective:**

To explore the correlation between parturients' uterine artery blood flow spectra in the first and second trimesters of pregnancy and fetal growth restriction (FGR).

**Methods:**

The data of parturients treated in our hospital from February 2018 to February 2020 were retrospectively analyzed, 50 parturients with FGR were selected as the FGR group, and other 50 healthy cases were selected as the control group. In the first trimester (11-12 weeks of gestation) and the second trimester of pregnancy (13–24 weeks of gestation), the parturients of the two groups accepted the color Doppler ultrasonography (CDS), their hemodynamics indicators of uterine artery were recorded, and the correlation between their uterine artery blood flow spectra in the two periods and FGR was analyzed with the Receiver Operating Characteristic (ROC) curve.

**Results:**

No statistical differences in the parturients' general information including age, gestational weeks, gravidity, and parity between the two groups were observed (*P* > 0.05); the newborn's body weight, Apgar scores, number of preterm infants, and the number of infants transferring to the neonatal intensive care unit (NICU) were significantly different between the two groups (*P* < 0.05); in the first and second trimesters of pregnancy, the uterine artery pulsatility index (UtA-PI), uterine artery resistance index (UtA-RI), maximal systolic flow velocity, and systolic/diastolic (UtA-S/D) ratio were significantly higher in the FGR group than in the control group (*P* < 0.05), and the time-averaged maximal velocity (TAMX) was significantly lower in the FGR group than in the control group (*P* < 0.001); in early pregnancy, the incidence of early diastolic notch at bilateral uterine arteries between the two groups was not significantly different (*P* > 0.05), and the unilateral and total incidence in the first trimester as well as the unilateral, bilateral, and total incidence in the second trimester were significantly higher in the FGR group than in the control group (*P* < 0.05); in the first trimester, the sensitivity of detecting FGR with a uterine artery blood flow spectrum was 0.820, AUC (95% CI) = 0.840 (0.757–0.923), and in the second trimester, it was 0.860, AUC (95% CI) = 0.900 (0.832–0.968).

**Conclusion:**

There is a correlation between uterine artery blood flow spectra in the first and second trimesters of pregnancy and FGR, and the sensitivity of spectrum in the first trimester is higher than that in the second trimester, presenting a better clinical application value.

## 1. Introduction

Fetal growth restriction (FGR) is one of the most common complications in the perinatal stage, and its diagnostic criteria are the failures of a fetus to achieve its due growth potential at a gestational age below the 10th percentile of the mean for that fetus of the same sex, or below 2,500 g after 37 weeks of gestation [1, 2]. Based on the different pathogenic causes, FGR has been clinically classified into two categories, namely, FGR of definite etiology due to maternal primary disease and pregnancy comorbidities and FGR of unknown etiology, also known as idiopathic FGR (IFGR), which accounts for about 40% of the total incidence of FGR [3–5]. FGR with a clear pathogenic cause can be eased after systemic treatment, while the effect of treating IFGR with measures such as nutritional support is limited, so most clinical studies focus on the prediction of IFGR [6–8]. However, regardless of the causative factors, FGR can improve the fetal mortality rate to 6–8 times that of normal perinatal infants [9], so early diagnosis and treatment are of great importance to improve the fetal prognosis.

Reviewing the previous literature, the sensitivity of the blood flow spectrum to predict IFGR has been demonstrated; to be specific, the middle cerebral artery (MCA) and fetal umbilical artery (FUA) are the first vessels to be affected at the onset of IFGR [10, 11], and the uterine artery, as the main way for the fetus to obtain blood supply from the mother, can also provide a basis for evaluating IFGR [12]. Compared with the MCA and FUA, the uterine artery blood flow spectrum can represent the hemodynamic relationship between the mother, uterus, and fetus more accurately, while the presence or absence of an early diastolic notch can also reflect the vascular resistance of the uterine artery [13, 14], which is associated with or higher than other arteries for FGR. Currently, most relevant studies have focused on the efficacy of diagnosing IFGR with uterine artery, but the correlation between the uterine artery blood flow spectrum and FGR remains unclear. Based on this, the association between uterine artery blood flow spectra in the first and second trimesters of pregnancy and FGR was explored herein, with the results reported as follows.

## 2. Data and Methods

### 2.1. Study Design

This retrospective study was conducted in our hospital from February 2018 to February 2020 to explore the association between uterine artery blood flow spectra in the first and second trimesters of pregnancy and FGR. It was a double-blind study, meaning that neither the research objects nor the researchers understood the trial grouping, and the study designer was responsible for arranging and controlling the full trial.

### 2.2. Research Object Enrollment

The data of parturients treated in our hospital from February 2018 to February 2020 were retrospectively analyzed, and the parturients were enrolled according to the following inclusion and exclusion criteria. Inclusion criteria: (1) the parturients were conceived naturally and were of singleton pregnancy; (2) the parturients were treated in our hospital the whole course and did not transfer to other hospitals in the middle of treatment; (3) the parturients did not have infection during pregnancy; (4) the parturients were free of severe pregnancy complications or comorbidities; (5) the parturients had no history of drinking or smoking; (6) the parturients were under the age of 35 years; (7) the fetus had no gross anatomical abnormalities and was determined to be chromosomally normal by amniocentesis; and (8) the clinical data of the parturients were complete. Exclusion criteria: (1) the parturients were unable to communicate with others due to hearing disorders, language disorders, unconsciousness, mental diseases, etc.; (2) the parturients quit the trial in the middle of the treatment; (3) the parturients were of multiple pregnancies; and (4) the clinical data of the parturients were missing.

Referring to the *Obstetrics and Gynaecology (9th Edition)* [15], the diagnostic criteria for FGR were the failures of a fetus to achieve its due growth potential at a gestational age below the 10th percentile of the mean for that fetus of the same sex.

### 2.3. Steps

Figure 1 shows the research steps.

A total of 100 parturients were enrolled in this study, 50 parturients with FGR were included in the FGR group, and the rest with healthy fetus were included in the control group. On the day that the parturients agreed to join the study, the study team collected the sociodemographic data and clinical performance data to establish the personal database; in the first trimester (11-12 gestational weeks) and second trimester of pregnancy (13–24 gestational weeks), color Doppler ultrasonography (CDS) was performed to all parturients to record their hemodynamics indicators and analyze their blood flow spectra; after delivery, the newborn body weight and Apgar scores were recorded, and the association between the uterine artery blood flow spectra of parturients in the first and second trimesters of pregnancy and FGR was analyzed with the Receiver Operating Characteristic (ROC) curve.

### 2.4. Moral Consideration

The study met the principles of the *World Medical Association Declaration of Helsinki* [16]. After enrollment, the study team explained the study purpose, meaning, content, and confidentiality to the parturients and asked the parturients to sign the informed consent.

### 2.5. Criteria for Quitting the Trial

For the patients with one of the following situations and who were judged by the study team as not suitable for continuously accepting the trial, their case record forms were reserved but not for data analysis: (1) those with severe pregnancy complications or comorbidities; (2) the subjects refused to proceed with the clinical trial in the process and proposed the demand to the study team of quitting the clinical trial.

### 2.6. Instruments and Methods

#### 2.6.1. Instruments

In the first trimester (11-12 gestational weeks) and second trimester of pregnancy (13–24 gestational weeks), CDS was performed to all parturients with the convex array probe of color Doppler ultrasonography (GE Voluson P6; NMPA (I) 20152062178), and the frequency was set as 1.0–5.0 MHz.

#### 2.6.2. Methods

The parturients lied down for rest for 10 min before the examination; then, in the spine position with a small amount of bladder filling, the CDS was performed by the abdomen. (1) Measurement of fetal biology parameters: the growth and development parameters of the fetus including biparietal diameter (BPD), head circumference, and abdominal circumference were measured to evaluate its development. (2) Steps of CDS: position the cervix, locally enlarge the image, move the probe to the junction of body of uterus and cervix on one side to show the upstroke of uterine artery and then obtain the uterine artery blood flow wave of 3 consecutive cardiac cycles, measure and record the uterine artery pulsatility index (UtA-PI), uterine artery resistance index (UtA-RI), and time-averaged maximal velocity (TAMX), calculate the systolic/diastolic (UtA-S/D) ratio with the internal software, then move the probe back to the cervix to measure the upstroke of opposite uterine artery, when measuring, set the width of CDS sampling gate to 2 mm and the angle between ultrasonic beam and blood flow to less than 30°, and record early diastolic notch in the first and second trimesters of pregnancy.

### 2.7. Observation Criteria

1. General information: the general information extract forms were established by the parturients themselves, covering inpatient number, name, age, gestational weeks, gravidity, parity, newborn body weight, Apgar scores [17], number of preterm infants, number of infants transferring to the neonatal intensive care unit (NICU), and place of residence, monthly income, and educational degree of the parturients
2. Blood flow spectra in the first and second trimesters of pregnancy: in the two periods, the UtA-PI, UtA-RI, and UtA-S/D indicators of the parturients in the two groups were compared
3. Incidence rates of early diastolic notch of the uterine artery: the incidence rates of early diastolic notch of the parturients in the two groups were calculated
4. Association between uterine artery blood flow spectra in the first and second trimesters of pregnancy and FGR: the association between UtA-PI, UtA-RI, and UtA-S/D in the two periods and FGR was analyzed with the ROC curve

### 2.8. Statistical Processing

In this study, the data processing software was SPSS20.0, the picture drawing software was GraphPad Prism 7 (GraphPad Software, San Diego, USA), the items included were enumeration data and measurement data, the methods used were the *X*^2^ test and *t*-test, and differences were considered statistically significant at *P* < 0.05.

## 3. Results

### 3.1. Comparison of Parturients' General Information

Between the two groups, the parturients' general information including age, gestational weeks, gravidity, and parity were not significantly different (*P* > 0.05), and the newborn body weight, Apgar scores, number of preterm infants, and number of infants transferring to the NICU were significantly different (*P* < 0.05), see Table 1.

### 3.2. Comparison of Parturients' Blood Flow Spectra in the Early Pregnancy and Pregnant Metaphase

In the early pregnancy and pregnant metaphase, the FGR group presented significantly higher UtA-PI, UtA-RI, and UtA-S/D (*P* < 0.05) and significantly lower TAMX (*P* < 0.001) than the control group, see Figure 2.

### 3.3. Comparison of Incidence Rates of Early Diastolic Notch of Parturients' Uterine Artery

In early pregnancy, the incidence rates of early diastolic notch of bilateral uterine arteries between the two groups were not significantly different (*P* > 0.05), and compared with the control group, the unilateral and total incidences in early pregnancy and unilateral, bilateral, and total incidences in the pregnant metaphase were significantly higher in the FGR group (*P* < 0.05), see Figure 3.

### 3.4. Correlation between Uterine Artery Blood Flow Spectra in the First and Second Trimesters of Pregnancy and FGR

The sensitivity of measuring FGR with the uterine artery blood flow spectrum in the first trimester of pregnancy was 0.820, AUC (95% CI) = 0.840 (0.757–0.923), and in the second trimester of pregnancy, it was 0.860, AUC (95% CI) = 0.900 (0.832–0.968), see Figure 4.

## 4. Discussion

FGR is a common obstetric complication with complex pathogenic factors, with macroscopic and microscopic pathological changes pointing to reduced blood flow resulting from the injury of blood vessels within the uterus-placenta, indicating that the uterine artery-fetus blood supply is an important factor affecting FGR [18, 19]. The uterine artery is an important artery that nourishes the fetus, which originates from the internal iliac artery. Its ascending branch gives off a tertiary artery in the uterine lining, and its terminal branch, the spiral artery, is widely distributed at the placental attachment. During normal pregnancy, nutrients of the parturient can be exchanged with the fetus through the intervillous spaces; from 3 gestational weeks, trophoblasts gradually erode and remodel uterine spiral arterioles, infiltrate into the vascular wall after 10 gestational weeks, and slowly extend to the decidua-uterus junction until vascular remodeling reaches its peak at 28 gestational weeks [20, 21]. Maternal physiologic changes during pregnancy can lead to widening of the caliber of the uterine spiral artery vessels and reduction of vessel resistance from high to low, thereby satisfying the blood supply to the placenta and allowing the fetus to obtain an adequate source of nutrients for growth and development. If the invasive potential of trophoblasts is not maintained because of comorbidities or other factors of the parturient during pregnancy, the process of erosion of the spiral arteries will consequentially be impaired, the invasion fails to reach its peak at 28 gestational weeks and extends only to the decidua, and the maternal spiral endometrial arteries exhibit degeneration of elastic fibers of the uterine wall, rendering elevated uterus-placenta resistance and an inability of the mother to supply blood to the fetus [22, 23]. To enhance blood supply, the general compensation for the mother is elevating uterine artery pressure, but high resistance, hypoxia, ischemia trigger contraction of uterine artery smooth muscle, and diastolic blood flow in the uterine artery cannot rise with gestational age, leading to the increased incidence of FGR. Therefore, the spectrum of blood flow in the uterine artery can reflect the variations of blood flow between the mother, uterus, and fetus and provide an objective basis for the clinical assessment of FGR.

In this study, no statistical differences in the parturients; age, gestational weeks, gravity, parity, and other general information between the two groups were observed (*P* > 0.05), but in the early pregnancy and pregnant metaphase, the FGR group obtained significantly higher UtA-PI, UtA-RI, and UtA-S/D (*P* < 0.05) and significantly lower TAMX (*P* < 0.001) than the control group, indicating elevated uterine artery resistance and reduced placental blood supply in the FGR group. Generally, the uterine artery resistance of normal pregnant women will continuously decrease as the gestational age increases, and both UtA-PI and UtA-RI should show a decreasing trend, and the fetus-placenta circulation will be significantly affected in a negative way when UtA-RI rises substantially. In the study by Jovian M. Wat et al., it was also confirmed that abnormal variations of UtA-PI and UtA-RI would trigger adverse outcomes such as IFGR [21]. Not only that but also the presence of high or low UtA-PI and UtA-RI affect the early diastolic notch of the uterine artery spectrum. The early diastolic notch occurs under high vascular resistance of the uterine artery and is not found under low resistance, so its incidence may also reflect the placental blood supply. This study showed that, in early pregnancy, the incidence of early diastolic notch at bilateral uterine arteries was not significantly different between the two groups (*P* > 0.05), and compared with the control group, the FGR group presented significantly higher unilateral and total incidences in early pregnancy and bilateral, unilateral, and total incidences in the pregnant metaphase (*P* < 0.05), indicating the sensitivity of the uterine artery blood flow spectrum in the pregnant metaphase was higher than that in early pregnancy, which might be due to the fact that, in the pregnant metaphase, the infiltration of trophocytes reached its peak while those with FGR presented low infiltration potential. Through validation with an ROC curve, it was found that the sensitivity of detecting FGR with the maternal uterine artery blood flow spectrum in the first trimester of pregnancy was 0.820, AUC (95% CI) = 0.840 (0.757–0.923), and in the second trimester of pregnancy, it was 0.860, AUC (95% CI) = 0.900 (0.832–0.968), demonstrating high correlation between uterine artery blood flow spectra in the two periods and FGR and that the sensitivity in the second trimester was better. It has been well established that FGR treatment before 30 weeks of gestation is most effective and brings little effect after 36 weeks of gestation [24], so it is extremely important to improve the detection rate of FGR in the first and second trimesters. In practice, the risk of FGR shall be evaluated by combining with the uterine artery blood flow spectra in the two periods, and early intervention measures shall be taken.

In conclusion, there is a correlation between uterine artery blood flow spectra in the first and second trimesters of pregnancy and FGR, and the sensitivity of detecting FGR with the spectra in the first trimester is higher than that in the second trimester, indicating a higher clinical application value.

## Figures and Tables

**Figure 1:** Research steps.

**Figure 2:** Comparison of blood flow spectra in the early pregnancy and pregnant metaphase ($\bar{\text{x}}$ ± *s*). *Note*. # indicated *P* < 0.05. (a) The blood flow spectrum in early pregnancy; the horizontal axis from left to right indicated UtA-PI, UtA-RI, and UtA-S/D, and the vertical axis indicated the blood flow spectrum; the black areas indicated the FGR group, and the gray areas indicated the control group. In the early pregnancy, the UtA-PI, UtA-RI, and UtA-S/D indicators of the FGR group were significantly higher than those of the control group (1.86 ± 0.67 vs. 1.39 ± 0.69, 0.74 ± 0.12 vs. 0.64 ± 0.10, and 3.92 ± 0.87 vs. 3.34 ± 0.88, *P* < 0.05). (b) The blood flow spectrum in the pregnant metaphase; the horizontal axis from left to right indicated UtA-PI, UtA-RI, and UtA-S/D, and the vertical axis indicated the blood flow spectrum; the black areas indicated the FGR group, and the gray areas indicated the control group. In the pregnant metaphase, the UtA-PI, UtA-RI, and UtA-S/D indicators of the FGR group were significantly higher than those of the control group (1.41 ± 0.96 vs. 0.98 ± 0.32, 0.70 ± 0.14 vs. 0.59 ± 0.13, and 3.12 ± 0.94 vs. 2.62 ± 0.68, *P* < 0.05). (c) The TAMX in the first and second trimesters of pregnancy; the horizontal axis from left to right indicated the two periods, and the vertical axis indicated TAMX (m/s). In both periods, the TAMXs were significantly lower in the FGR group than in the control group (0.24 ± 0.11 vs. 0.57 ± 0.12 and 0.37 ± 0.12 vs. 0.65 ± 0.15, *P* < 0.001).

**Figure 3:** Comparison of incidence rates of early diastolic notch of parturients' uterine artery [*n*(%)]. The horizontal axes from left to right indicated bilateral, unilateral, and total incidences, and the vertical axis indicated the cases with early diastolic notch; the black areas indicated the FGR group, and the gray areas indicated the control group. # meant *P* < 0.05. (a) The early diastolic notch of the uterine artery in early pregnancy, no significant difference in bilateral incidence between the FGR group and control group was observed (20 vs. 21, *P* > 0.05), and the unilateral and total incidences were significantly higher in the FGR group than in the control group (21 vs. 10 and 41 vs. 31, *P* < 0.05). (b) The early diastolic notch of the uterine artery in the pregnant metaphase, and the bilateral, unilateral, and total incidences were significantly higher in the FGR group than in the control group (25 vs. 3, 12 vs. 2, and 37 vs. 5, *P* < 0.05).

**Figure 4:** Correlation between uterine artery blood flow spectra in the first and second trimesters of pregnancy and FGR.

**Table 1:** Comparison of parturients' general information.

Group	FGR group (*n* = 50)	Control group (*n* = 50)	*X* ^2^/*t*	*P*
*Age (years)*				
Range	22–34	21–34		
Mean age	28.65 ± 2.50	28.72 ± 2.41	0.143	0.887
Gestation (weeks)	12.10 ± 1.68	12.13 ± 1.57	0.092	0.927
Gravidity (times)	2.21 ± 0.32	2.15 ± 0.30	0.967	0.336
Parity (times)	1.00 ± 0.21	1.05 ± 0.23	1.135	0.259
Newborn body weight (g)	1,921.65 ± 254.20	3,410.68 ± 421.68	21.384	<0.001

*Apgar scores*				
1 min	7.64 ± 0.68	9.02 ± 0.45	11.967	<0.001
5 min	8.21 ± 0.48	9.46 ± 0.58	11.740	<0.001
10 min	8.38 ± 0.68	9.72 ± 0.46	11.541	<0.001
Number of preterm infants	18	4	11.422	0.001
Number of infants transferring to the NICU	17	3	12.500	<0.001
Place of residence of the parturient			0.041	0.841
Urban area	28	27		
Rural area	22	23		
Family monthly income (Yuan)			0.170	0.680
≥4,000	30	32		
<4,000	20	18		
Educational degree			0.040	0.841
Senior high school and below	26	27		
College and above	24	23		

## Data Availability

Data to support the findings of this study are available on reasonable request from the corresponding author.
